The article "Development of mucus-penetrating iodine loaded self-emulsifying system for local vaginal delivery" was published in 2022. Journal: PLoS One.

# Development of mucus-penetrating iodine loaded self-emulsifying system for local vaginal delivery

**DOI:** 10.1371/journal.pone.0266296

**Published:** 2022-03-31

**Authors:** Saima Fida, Aamir Jalil, Rukhshanda Habib, Muhammad Akhlaq, Arshad Mahmood, Muhammad Usman Minhas, Kifayat Ullah Khan, Asif Nawaz

**Affiliations:** 1 Faculty of Pharmacy, Department of Pharmaceutics, Gomal University, Dera Ismail Khan, Pakistan; 2 Faculty of Pharmacy, Department of Pharmaceutics, Bahauddin Zakariya University, Multan, Pakistan; 3 College of Pharmacy, Al Ain University, Abu Dhabi Campus, Abu Dhabi, United Arab Emirates; 4 AAU Health and Biomedical Research Center, Al Ain University, Abu Dhabi, United Arab Emirates; 5 College of Pharmacy, University of Sargodha, University Road Sargodha City, Punjab, Pakistan; 6 Quaid-e-Azam College of Pharmacy, Sahiwal, Punjab, Pakistan; ISF College of Pharmacy, Moga, Punjab, India, INDIA

## Abstract

The major goal of this project was to formulate iodine-based self nano-emulsifying drug delivery system to provide improve antimicrobial activity and enhanced mucosal residence time via mucus penetration. Iodine SNEDDS (Self nano-emulsifying drug delivery system) with different concentration were formulated using castor oil as the oil phase, cremophor ethoxylated (CrEL) as a surfactant and after screening a number of vehicles, PEG 400 was employed as co-surfactant. Self-emulsification time, thermodynamic stability tests, robustness to dilution, percent transmittance, droplet size, and drug release were measured. Ternary phase diagrams were plotted to determine the area of emulsification. When compared to the commercial formulation, dissolving experiments revealed that the iodine from the SNEDDS enhanced aqueous solubility. *In-vitro* iodine release was determined to be around 15% per hour, with muco-adhesive and, muco-penetrating characteristics showing a 38-fold improvement. Furthermore, SNEDDS demonstrated significant antibacterial efficacy against Escherichia coli and Staphylococcus aureus. Similarly, when compared to marketed drugs, *in-vitro* drug absorption profile from the manufactured SNEDDS shown to be much higher. According to these results iodine containing SNEDDS could be a useful new formulation for iodine mucosal usage.

## Introduction

The pathogenic microorganisms like bacteria, viruses, protozoa and fungi can play a major role in the development of many pathogenic infections by their colonization in the mucosal tissue [1]. To treat such pathogenic infections, antibiotics or antiseptics are commonly used. However, it is observed that due to irrational use, antibiotics are more prone to microbial resistance. Due to the low risk of developing resistance and multiple mode of action, antiseptics and disinfectants are found to be a suitable alternatives of antibiotics for the prevention and treatment of mucosal infections [2].

Iodine is a well-known powerful and highly effective disinfectant which has not only broad-spectrum antimicrobial activity against bacteria, fungi, protozoan, bacteriophages, spores and certain viruses, but is easily available and relatively inexpensive [3,4]. Its work on the principle of immediate penetration into microorganism by binding to proteins and enzymes by altering phospholipid membrane structure leading to rapid cell death [5]. The major advantage of using iodine as bactericidal because it irreversibly damages the bacterial cell and has found no tendency to cause resistance. The main side effects of iodine include pain, irritation and skin staining [4].

Iodine due to its low aqueous solubility, from the drug delivery point of view, its application as antimicrobial agent is challenging. In order to increase iodine concentration in formulations, alcoholic iodine solutions also have been used for a long time. A povidone–iodine complex which is a stable complex of iodine and polyvinylpyrrolidone (PVP) was developed as antiseptic agent [4]. The PVP have iodophor property [5], it is a water soluble and biocompatible polymer [6]. In povidone–iodine complex, all iodine is entrapped between two carbonyl groups of PVP and tri-iodide anion through hydrogen bonds and free iodine concentration in solution is generally found very low [7]. As antimicrobial effect of povidone–iodine complex is greatly dependent on release of iodine from the complex and this release of iodine cannot be controlled. Moreover, PVP is only poorly biodegradable [6].

In addition, iodine only remains on mucosal membranes for a short time due to lack of any muco-adhesive properties [4]. Due to high vapor pressure, inactivation in living tissues and susceptibility to evaporation, the concentration of freely available active iodine which possibly found less than desired activity when administered *in-vivo*. In order to overcome the shortcomings of current formulations, it was the objective of this work to develop iodine formulations providing a controlled drug application and a prolonged mucosal residence time.

So, to gain required concentration in the cervical-vaginal side, it will be favorable to distribute iodine concentration in a constant way. Restrictions like leakage from the cavity and low residence time are reported in conventional vaginal drug delivery system which results in discomfort, poor patient compliance and result in a decrease in therapeutic efficacy [8]. In vaginal drug delivery system to achieve therapeutic activity, the dose of a drug is greater than required dose. Mostly marketed vaginal tablets have 200 mg povidone iodine per unit dose, while semisolid have 2% w/w povidone iodine. A great interest in innovative vaginal drug delivery methods has been noted recently with a focus to improving drug solubility, bio-availability, bio-adhesion and sustained release. The bio-adhesive dosage forms with sustained release behavior have advantages such prolonged and constant retention of drug concentration locally at desired position. As a result of the reduction in dosing frequency, the patient compliance has improved.

Nanotechnology has shown great potential for biomedical applications because of their tunable physicochemical properties especially bio-compatibility, improved solubility and bioavailability of poorly soluble drugs [9–14]. The significance and main objective of the present work is to enhance the solubility of poorly-water soluble therapeutic agents & to develop muco-adhesive based vaginal SNEDDS for iodine which will be capable of spreading & penetrating in the mucus layer.

## Material and methods

### Chemicals/Materials

Elemental iodine, Povidone-iodine, (from pharmaceutics department faculty of pharmacy), Tween-80, tween-20, tween-85 Cremophor EL, PEG 400, Ethanol. The elemental iodine was tested for identification and utilized exactly as it was given to us. Chemicals and reagents were bought from a variety of commercial sources and were of analytical grade for buffer synthesis, analytical solution preparation, and other general experimental objectives.

### Solubility studies

Solubility studies of iodine in different excipients like oils, surfactants and co-surfactant was carried out with the help of shake flask method. For this purpose an extra concentration of drug (iodine) was incorporated in the each utilized excipient. The resultant mixture was properly vortexed for 30 seconds to achieve homogeneous combination. The resultant mixtures were properly shaken for 50 strokes/minute, at 30°C for 48 hours followed by a 24 hours period of balance in a water bath. After that prepared mixture were subjected to centrifugation for 10 minutes at 3000 rpm. The supernatant layer of solution was collected from each resultant mixture and then passed via Millipore filter membrane (0.45 μ). UV visible double beam spectrophotometer (Shimadzu UV Spectrophotometer) was used to quantify iodine in each sample at 225 nm using ethanol as blank solution.

### Preliminary screening of surfactant and co-surfactant

The emulsification time and percentage transmittance of several surfactants and co-surfactants were used to further screen them. In 300 mg of selected oil phase, 200 mg of surfactant and 100 mg of co-surfactant was properly mixed. The resultant mixture heated to 50 degrees Celsius. To measure emulsification efficiency, the number of flask inversions were calculated.

### Construction of pseudo ternary phase diagram

To construct the ternary phase diagram excipients with various ratios has been used. Each peak of ternary phase diagram denotes the every component of isotropic mixture. The phase behavior of each excipient was determined by varying amount of each component by maintaining HPMC concentration constant. The mixture composition was evaluated for self-emulsification characteristics. At 37°C, the SNEDDS mixture (1 ml) was properly dispersed in 100 ml of deionized water. Resultant mixture was also subjected to percentage (%) transmittance, poly dispersity index (PDI) and the droplet size determination.

### Preparation of SNEDDS

SNEDDS formulations were formulated with different concentration of oil (20–30%), surfactant (40–60%) and solvent/co- surfactant (10–20%). A single unit dose of iodine with various strength (2 mg, 3 mg, 4 mg and 5 mg) was added in all formulations as shown in Table 1. In glass vials the preparations were formulated by proper properly mixing the drug (iodine) into oily phase properly by the addition of surfactant and co-surfactant. The total mass of the formulations was kept constant. The resultant mixture were mixed continuously. To obtain a homogeneous isotropic mixture, vortex mixing and sonication for a few minutes are used. The SNEDDS formulations were kept at room temperature for future use.

**Table 1:** SNEDDS formulations comprises of different concentration of oils, surfactant and co-surfactants.

Formulations	surfactant co-surfactant ratio (Km ratio)	Oil Castor oil (%w /w)	Surfactant Cremophor EL (%w/w)	Co-surfactant PEG 400 (%w/w)	Iodine (%w/w)	HPMC (% w/w)
F1	1:1	25	36.75	36.75	1	0.5
F2	1:1	30	34.25	34.25	1	0.5
F3	1:1	35	31.75	31.75	1	0.5
F4	2:1	25	49	24.5	1	0.5
F5	2:1	30	45.67	22.83	1	0.5
F6	2:1	35	42.34	21.17	1	0.5
F7	1:2	25	24.5	49	1	0.5
F8	1:2	30	22.83	45.67	1	0.5
F9	1:2	35	21.17	42.33	1	0.5
F10	2:1	30	45.67	22.83	1	0.5
F11	2:1	30	45.34	22.66	1.5	0.5
F12	2:1	30	45	22.5	2	0.5

### Characterization of SNEDDS

#### Physicochemical evaluation of SNEDDS

*Percentage (%) transmittance*. 1 ml of each SNEDD formulation was 100 times diluted in distilled water. Percentage (%) transmittance was evaluated by using the double beam UV -Visible spectrophotometer (shimadzo, Bioequivalence) at 255 nm [15].

*Dispersibility test*. In order to determine the self-emulsification properties of SNEDDS on magnetic hot stirrer plate (Gomal University) the dispersibility test was conducted. 1 ml of optimized SNEDDS was properly dispersed in 100 ml of deionized water at 50 rpm and at 37°C temperature. The time taken by SNEDDS to form complete dispersion into a clear, transparent dispersion was recorded [16].

*Saturation solubility*. The shaking flask method was utilized to determine the saturation solubility of optimized SNEDDS [17]. Excess amount of Iodine was mixed in 1 ml of optimized SNEDDS (F6, F10 and F11) and mixed for 10 minutes by vortex machine. Subsequently, resultant mixture was properly standardized at temperature of 37°C for 48h at 50 rpm in water shaking bath (WNB -7, Memmert, Buchenbach, Germany).

*Visual observation for self-emulsification*. A visual assessment were carried out in order to observe the self-emulsification characteristics (Talegaonkar et al). A single dose 2 mL of formulation was added to 250 ml of distilled water in a glass beaker and kept at a temperature of 37 ± 0.5°C. Then the mixture was mixed gently and properly with the help of magnetic stirrer. The ability to spontaneously emulsify and emulsion droplet progress was measured. Depending on the SNEDDS appearance, the time needed for its emulsification and dispersibility SNEDDS were also categorized [18].

*Drug content*. Prepared SNEDDS containing 1% iodine was added in 50 ml volumetric flask containing ethanol and properly mixed by shaking or inverting the volumetric flask 2–3 times. 0.1 ml of this solution was diluted with 25 ml fresh ethanol and by using the UV-spectrophotometer the drug content was determined at 255 nm.

*Phase separation study*. 0.05 ml of each SNEDDS was added to glass test tube which having 5 ml of 0.1 N HCl and double distilled water. Each mixture was stored for 2 hours after inverting the test tube 3–4 times and also observed visually for any phase separation.

*Viscosity determination*. At 25°C, viscosity of the optimized SNEDDS was determined using a Brookfield viscometer. The spindle size employed in this investigation was 31s. The rotational speed was kept at 40 rpm. The viscosity was measured in centipoises (cP) and the procedure was performed three times.

*Thermodynamic stability testing*. The prepared formulations were further subjected to thermodynamic stability testing. So prepared formulations were stored in fridge (PEL refrigerator) at 4°C and then stored at 50°C in an incubator (Panasonic). Those formulations passing these tests successfully were then subjected to Freeze thaw cycles [19].

*Freeze thaw cycle*. For the formulations, freeze-thaw cycles between -21°C and +25°C were investigated, having storage conditions at each temperature for at least 48hours.First formulation was stored in Haier thermo cool HF 240T Freezer (HPZ Nigeria) at -21°C and then kept in an oven at 25°C.Those formulations which were passed through these thermodynamic stress testing were father subjected to centrifugation test which was followed by dispersibility test in order to evaluate the efficiency for self-emulsification and /or robustness to dilution.

*Centrifugation test*. Sample were centrifuged at speed of 3500 rpm on centrifuge machine (EBA 20, centrifuge, Germany) after being properly diluted 100 times with distilled water for half an hour and for any phase separation examined visually.** **

*Self-emulsification time*. In order to determine the efficiency of self-emulsification, the rate of emulsification was considered as a major indicator. The SNEDDS which was subjected to slight agitation should disperse quickly and completely [20].

*Cloud point measurement*. This test was conducted on optimized iodine SNEDDS formulations which were hundred folds diluted with distilled water. After that kept on a water bath. This cloud point of diluted SNEDDS formulations was evaluated by temperature at which any sudden change observed in physical appearance i.e. cloudiness seemed. The water bath temperature was raised at a degree of 5°C per min. Temperature was noted by using thermometer [21].

*Robustness to dilution*. This study of iodine containing SNEDDS were conducted by dilution method by using 50, 100, and 1000 times dilution through different media of dissolution such as water, pH 1.2 buffer and pH 6.8 buffer. The diluted SNEDDS formulations were kept for 12hrs. Especially noticeable for any drug precipitation or phase separation [22].

*Droplet size*, *zeta potential and poly dispersity Index (PDI)*. Optimized SNEDDS formulations were 100 times diluted with de-ionized water and properly homogenized with the help of Ultrasonic Homogenizer (E60 H, Elma Hans Schmid Bauer & Co, Singen, Germany) for 5 minutes [23,24]. Optimized SNEDDS formulation were further evaluated for droplet size, Zeta -potential and polydispersity index with by using Zeta sizer (ZS90, Malvern instrument, London, UK).

*Scanning electron microscopy (SEM)*. In order to determine the morphological characteristics of optimized SNEDDS formulation (F11), scanning electron microscopy (SEM) (S-4100, Hitachi, Japan) analysis was carried out at 15 keV accelerating voltage.

*Fourier transform infrared spectroscopy (FTIR)*. The compatibility of the drug with the various excipients used in the formulations was assessed by Fourier transform infrared spectroscopy. Iodine, Cremophor EL, Tween-80, Castor oil, PEG 400 and formulation. All the samples were analyzed in the range of 4500–450 cm^-1^. Zinc selenium ATR (attenuated total 58 reference) mode fixed at 16 scans per sample was used for the analysis of samples [25].

#### Antimicrobial activity of SNEDDS

To determine the antimicrobial activity, iodine loaded SNEDDS was associated for 8 hrs. Gram negative E. coli was utilized as a model germ in this investigation, having a bacterial density of roughly 3.0 108 CFU/mL in LB medium (1 McFarland). 250 liters of 1 McFarland bacterial suspension were mixed 1:1 with 250 liters of LB medium/water mixture, providing a final bacterial density of 1.5 108 CFU/mL. In one sense, SNEDDS containing 1% iodine were diluted 1:40, while 111g of free iodine was correctly dissolved in 500 mL of growth media so get 125 g/mL iodine. Controls included SEDDS without iodine and growth medium without iodine. As a blank, LB medium was used without any drugs or bacteria. The samples were kept in a thermo-mixer set to 37degrees Celsius and 600 rpm. At a certain period, aliquots (100 L) where Optical density was measured at 600 nm using a micro-plate reader after being transferred to a 96-well plate. At each time point, without medicine, the bacterial population in LB medium was found to be 100%.

### *In-vitro* evaluation of muco-adhesive characteristics of SNEDDS

The iodine and iodine containing SNEDDS were evaluated for their muco-adhesive properties fluorescent labeled by integration of FDA for the evaluation of mucoadhesive characteristics. So, for this purpose freshly slaughtered vaginal mucosa from a local slaughter house was collected [26]. First of all vagina was properly cleaned and washed with 100 mM phosphate buffered saline pH 6.8. Afterward, the small cut pieces 4 ×2 cm of mucosal tissue was organized and properly fixed on half cut falcon tubes that had already been positioned at a 45 degree angle in a 37°C incubation chamber. Then the small pieces of mucosal membrane were continuously washed with phosphate buffer pH 6.8 at a flow rate of 1 ml/min for 5 min. In next step 30 mg of iodine samples were placed separately on each mucosa for 10 min to get properly adsorb on the surface and then phosphate buffer flow was restarted at a constant flow rate of 1 ml/min. Phosphate buffer flowing down the mucosa was gathered at predetermined time points like 30 min, 60 min, 90 min, 120 min, 150 min and 180 min. For control sample, phosphate buffer (100 mM, pH 6.8) flowing down the mucosa deprived of any iodine was gathered. 30 mg of iodine were dissolved in it and used to calculate the percentage of iodine left on mucosa. To quantitatively hydrolyze iodine to sodium fluorescein, all the collected samples were properly treated with equal volume of 5 M NaOH. The samples were incubated at 37°C for 10 minutes while stirring continuously, and then centrifuged for 5 minutes at 13400 rpm. Finally, a micro plate reader was used to transfer 100 l of each sample to a micro plate. (M-200 spectrometer; Tecan infinite, Grodig, Austria) and fluorescence force was measured at an emission wavelength of 225 nm and exciting wavelength of 485 nm [27].

### *In-vitro* iodine release studies

*In-vitro* release of iodine from SNEDDS was quantified via iodometric method. Briefly, 3 mg of SNEDDS containing iodine and iodine (5 mM) were applied to intestinal mucosal membrane and was incubated for 5 min at 37°C letting adhesion to take place. After proper fixing mucosa on cylinder with the help of glue, 3 ml of phosphate buffer (100 mM, pH 6.8) was filled above mucosal tissue and incubated for 3 h at 37°C. After every 30 minutes, a total of 100 l of samples were withdrawn. and were replaced with same volume of buffer maintained at 37°C. Filtration of samples were carried out by using 0.45 μm membrane filter and iodine released was quantified by method of UV Spectrophotometry. On a UV spectrophotometer, a UV-Vis scan of iodine in the presence of potassium iodide (5 percent w/v initially) was reported over a range of 200 nm to 800 nm (Shimadzu 1800). Absorbance with λ max at 255 nm.

### Statistical analysis

Statistical analysis were conducted by using the ANOVA, one-way analysis of variance followed a statistical significance value of less than 0.05 using student t-test. After performing all of the trials in triplicates, the data were displayed as mean SD.

## Results

### Solubility studies

The solubility of iodine was checked in various oils, castor oil, cajuput oil, turpentine oil, olive oil, cinnamon oil, orange oil and peppermint oil, surfactants like Cremophor EL, cremophor RH, Tween-85, Tween-80, captex-300 and Tween-20 and co-surfactants like PEG 400, Propylene glycol, polyethylene glycol.The data shown in the Fig 1. Among all screened oils, iodine exhibited maximum solubility in castor oil found to be 67.6 ± 0.577 mg/mL, followed by cajuput oil (37.0 ± 78) mg/mL, while the least solubility was observed with peppermint oil found to 6.21 ± 0.57 mg/mL as shown in Fig 1. Based on the above-mentioned results, the castor oil, selected as oil phase for more studies. The surfactant and co-surfactant were also selected depending on their capability to fairly solubilize iodine that was found to be ranging from 99 ± 43 mg/mL, 80 ± 78 mg/mL, 62 ± 28 mg/mL, 53 ± 75 mg/mL, 45 ± 66 mg/mL for Cremophor EL, cremophor RH, Tween-85, Tween-80, captex-300 and Tween-20, respectively as depicte in Fig 2. The co-surfactant was also selected on the basis of their ability to solubilize iodine that was found to be ranging from 380 ± 72 mg/mL, 98 ± 58 mg/mL and 74 ± 71 mg/mL for PEG 400, Propylene glycol, polyethylene glycol respectively depending on their ability to solubilize iodine as shown in Fig 2.

**Fig 1:** Solubility studies of iodine on different oils.

**Fig 2:** Solubility studies of iodine in different surfactants.

### Preliminary screening of surfactants

Cremophor EL, Tween-80 and Cremophor RH were nominated for the investigation of emulsification properties as they having satisfactory emulsifying ability for iodine. Castor oil was added in the selected surfactant having ratio 1:1 and the resulting mixture 50 mg was made diluted upto 50 mL, percent transmittance values of the different dispersions were attained using distilled water as 97.7 ± 0.61, 84.3 ± 1.13 and 85.4 ± 0.99 with chromophore EL, Tween-80, Cremophor RH and PEG 400 as the surfactants respectively.

### Preliminary screening of co-surfactants

In this work PEG 400, the present study PEG 400, propylene glycole and polyethylene glycol was studied as the co surfactant in order to improve the emulsification capability of Cremophor EL. The percentage (%) transmittance values ofdifferent dispersions were found to be 99.3 ± 0.55, 98.9 ± 0.18 and 87.3 ± 1.74 with PEG 400, Propylene glycol, polyethylene glycol respectively as the co-surfactant.

### Pseudoternary phase diagram

To construct pseudoternary phase diagram ternary mixture were prepared by utilizing the formulation excepients with the main aim having maximum solubilizing capability for iodine. Based on the clarity and on % transmittance, the ternary mixture were characterized as a bad or a good emulsion.By changing concentration of excipients like oil, surfactant and co-surfactant different formulations were formulated and emulsification time, % transmittance, and a clarity test, poly desperity index and droplet size were all evaluated. The results of all prepared formulations are shown in Table 2. The formulation having clear appearance and having percentage transmittance value of equal or greater than 85% were suggested as”good emulsion”. Outcomes of the experiment showed the area of transparent emulsions clearly with pseudo-ternary graph (Fig 1). SNEDDS preparation used a variety of Km ratios (surfactant to co-surfactant ratios).

**Table 2:** Composition of SNEDDS containing Iodine with thermodynamic stability indicators.

				Thermodynamic stability test			
Formulations	Percentage Transmittance	Emulsification time (sec)	Visual observation	Centrifugation	Heating cooling	Freeze thaw cycle	Cloud point
F1	79.2	38	Turbid	NPS	**Stable**	NC	**NC**
F2	88	19.15	Transparent	NPS	**stable**	NC	**NC**
F3	79.5	29	Turbid	NPS	**stable**	**NC**	**NC**
F4	85.2	21	transparent	NPS	**stable**	NC	**NC**
F5	82.1	24	slightly clear	NPS	**stable**	NC	**NC**
F6	93	15	transparent	NPS	**stable**	NC	**NC**
F7	85.25	18	transparent	NPS	**stable**	NC	**NC**
F8	83.5	25	slightly clear	NPS	**stable**	NC	**NC**
F9	77.9	21.5	Turbid	NPS	**stable**	NC	**NC**
F10	91	14.6	transparent	NPS	**stable**	NC	**NC**
F11	89	18	transparent	NPS	**stable**	NC	**NC**
F12	77.3	28	Turbid	NPS	**stable**	NC	**NC**

### Preperation of SNEDDS

Twelve formulation of SNEDDS were prepared according to composition depicted in Table 1. All formulation were evaluated for different parameters as shown in Table 2. The SNEDDS preperations which were screened out from phase behavior study further exposed to various stress condition such as heating and cooling cycle, centrifugation testing and freez thaw cycle. The results are shown (Table 2). The transmittance (%T) measures the transerancy and clarity of nano-emulsion [28]. Formulations F6, F10 and F11 exhibited maximum % transmittance value 93%, 91% and 89% respectively and found transparent and satisfactory (Table 2) and then were subjected to further studies.

Dispersibility characteristic of SNEDDS depends the upon the degree to surfactant lessens the interfacial tension at oil-water interface. In aqous media after 10, 100, and 1000 times dilution, all of the SNEDDS formulations form a fine nano emulsion having no phase separation or coalescence and found clear. Table 2 showed percent transmittance, cloud point results and Table 3 showed the saturation solubility for all iodine-containing SNEDDS.

**Table 3:** Zeta potential and average size of oily droplets of Iodine SNEDDS.

Formulation	Z. average (d.nm) ± SD	PDI± SD	Zeta potential (mV) ± SD	Saturation solubility mg/ml	viscosity (cp) ± SD
F6	359.5±4.04	0.368±1.10	-16.2 ± 0.301	10.04 ± 0.08	94.70 ± 1.38
F10	338.3±3.67	0.8±2.12	-7.58 ± 0.410	9.1 ± 0.12	74.25 ± 1.11
F11	233.8±4.76	0.446±3.01	-19.7 ± 0.342	10 ± 0.2	84.32 ± 1.67

### Droplet size, PDI, and zeta potential determination

Results of study revealed that formulation F11 showed lowest droplet size (233 ± 5.54 nm) having poly dispersity index (PDI) of 0.44 ± 0.012 and displaying a consistent size distribution which were subjected to further studies as shown in Table 3.

The zeta potential of the optimized SNEDDS formulations F6, F10 and F11 was found to be -16.2, -7.58 and -19.7 mV respectively as shown in Table 3 which complies with the requirement of the zeta potential for particle stability. The viscosity of the optimized SNEDDS were determined. The viscosity of F11 was found to be 84.32 ± 1.67 cP. The lesser visosity of F10 compared to F6 and F11 which may be due to the greater co-surfactant amount as shown in Table 3.

### Characterization of SNEDDS

Selected SNEDDS formulations were exposed to thermodynamic stability testing by keeping them at tempersture of 4°C in a refrigerator and 50°C in oven, properly observed visually. They were graded on a scale after a visual evaluation. Table 2 shows the results of thermodynamic stability testing. freeze-thaw cycles that occur between -21°C and +25°C kept at storage condition at each temperature for not less than 48hrs were calculated for the selected formulatons. After each cycle, formulations were recognised and visually evaluated, as shown in Table 2. Selected formulations were centrifuged centrifuge machine (EBA 20, centrifuge, Germany) at 3500 rpm, after 30 minutes of being diluted 100 times with distilled water. This measurement is a vital indiactor for SNEDDS formulations which was formulated from non ionic surfactans. Robustness to dilution of Iodine containing SNEDDS was performed by diluting with 50, 100 and 1000 folds by different media for dissolution such as water, pH 3.8 buffer solution, and pH 4.8 buffer solution. Droplet size distribution have a key part for the evaluation of self nanoemulsifying system. The size of the droplets is thought to be related to drug absorption, as evidenced by earlier research. The smaller the droplet size of the formulation, more will be the surface area available for drug absorption. Droplet size and PDI of developed formulations (F6, F10 and F11) are shown in Table 3.

### Scanning electron microscopy (SEM)

SEM images of diluted optimised formulation (F11) at different magnification is shown in Fig 3. Particles were found spherical and the droplet size was found to be around 150–200 nm having size distribution similar to the results obtained by zetasizer.

**Fig 3:** SEM images of SNEDDS formulation at different magnifications.

### Interaction studies by fourier transform infrared spectroscop

The interaction studies of the iodine (drug), formulation components, optimized formulation (F11) were analyzed by the FTIR as shown in Fig 4. Stability of iodine and its compatibility with the excipients was confirmed by the comparison of IR spectra of pure drug with formulation components. The FTIR pectrum of pure iodine drug exhibited the absorption peaks at 2925 cm^−1^ and 2562 cm^−1^ because of iodide group. The SNEDDS formulation characteristic peaks i.e., 3474.98 cm^−1^, 2924.47 cm^−1^, 1740.79 cm^−1^ were held in the FTIR pectra of SNEDDS along with all excepients having no exra peaks. This FTIR finding suggested that there was no interaction or compatibility between iodine containg SNEDDS, formulation excepients and the drug.

**Fig 4:** FTIR Spectra of (A) PEG 400, (B) Cremophor EL (C), castor oil (D), Iodine, (E) HPMC and (F) Iodine SNEDDS.

### *In-vitro* evaluation of muco-adhesive properties

Results of *in-vitro* muco-adhesive studies conducted on vaginal mucosa is illustrated in Fig 5 which showed that SNEDDS containing iodine complex is higher mucoadhesive than the simple -iodine. As its elucidated from the results that mucoadhesive properties of SEDDS containing iodine were 38-fold improved as compared with simple iodine. Almost 38% of SEDDS containing iodine remained attached to the mucosal membrane after 3 hours. Iodine release from SEDDS-iodine, unmodified iodine and unformulated iodine/controlled formulation as control applied to freshly excised vaginal mucosal surface for a time period of 3 hrs.

**Fig 5:** Iodine release as a function of muco-adhesion and muco-penetration from oily droplets of SNEDDS.

### Antimicrobial activity of SNEDDS

The antimicrobial activity of iodine containing SNEDDS was compared with simple iodine. The results shown that iodine containing SNEDDS formulation (1%) have enhanced antimicrobial activity when compared with simple iodine over a time period for 8 hours. The results shown that the ability of bacterial cells to survive which was gound reduced to 1/3 in case of iodine containing SNEDDS formulation (1%) within the first 2 h while simple iodine showing 59% viability as shown in Fig 6. After 8 h, SNEDDS showed 2-fold enhanced antimicrobial activity in copmarision to simple iodine as shown in Fig 6.

**Fig 6:** Percentage viability of microorganisms over the time period of 8 hrs.

### *In-vitro* iodine release studies

#### Quantification of iodine in the complex by iodometric titration

Percentage of iodine loaded in complex was quantified as described by Wang et al. with slight modifications [29]. In short, 0.1 g of SNEDDS containing iodine complex was properly was dissolved in 4ml of ethanol. Thereafter, 10 ml of demineralized was added and titrated against 0.01 M standard solution of Na2S2O3. Titration was carried out until continued until the colour of solution changed into light-yellow color. Then 1 ml 0.5% w/v starch solution was mixed as starch–iodine indicator to turn the solution blue. Titration was stopped until a colorless solution appeared as the end point. Each sample was titrated three times The iodine [%] in complex was calculated with the help of following equation.

$$\text{Iodine}\;\left[\%\right]=0.1269\times \frac{CNa2S2O3\times VNa2S2O3}{m}\times 100$$

Where, C_Na2S2O3_ represents the sodium thiosulfate standard solution concentration, V_Na2S2O3_ is the volume of ‘Sodium thiosulfate’ standard solution mixed while during titration (ml),while ‘m’ shows the weight (gram) of iodine containg SNEDDS. The percentage of iodine released from iodine containing SNEDDS were applied to freshly excised porcine intestinal mucosa. After 3 hours, almost 44% of iodine was released from the iodine containing SNEDDS as compared with 95% from unmodified Iodine. By contrast, iodine used as control released almost 90% within an hour as shown in Fig 7.

**Fig 7:** Iodine release from oily droplets of SNEDDS over the time period of 7 hrs.

## Discussion

For stable SNEDDS formulation, solubility of drug in lipid excipients considered as an important parameter which further cause efficient drug loading. Identifying the appropriate oil, surfactant and co-surfactant with maximum solubilizing capability for drug, not to mention to attains loading of drug at optimum capacity but minimize the final volume of the SNEDDS too [30]. The investigation properly discriminated the capability of the surfactants to emulsify the already selected oily phase, indicating that cremophor EL had the best emulsifying performance of all the surfactants tested. As a result, cremophor EL was chosen as a surfactant for further investigation. Turbidimetry tests were also carried out to see how well different surfactants emulsified the chosen oil phase, castor oil. It was crucial to see if the oil-surfactant mixture could disperse well enough to generate a spontaneous micro-emulsion before using it in SNEDDS formulations [31]. Propylene glycol, polyethylene glycol respectively as a co-surfactant, it was observed that both PEG 400 and propylene glycol found to be equivalent in emulsifying castor oil when mixed with Cremophor EL. As a result, the findings from the solubility investigations, as well as the well-known potential of PEG 400 as a co-surfactant were taken into account for formulation design [32].

The formulation having clear appearance and having percentage transmittance value of equal or greater than 85% were suggested as “good emulsion”. Outcomes of the experiment showed the area of transparent emulsions clearly with pseudo-ternary graph (Fig 8). SNEDDS preparation used a variety of Km ratios (surfactant to co-surfactant ratios). The surface area of clear emulsions with km ratios of 1:1, 2:1, and 1:2, respectively is shown in (Fig 8A–8C), with the amount of castor oil changing from 15 to 35 percent for each km ratio. In the formulation of SEDDS, the dotted component the number of clear emulsions generated by using relevant km ratio with oil.km ratio of 2:1 area showed larger area and found transparent emulsion. The main aim of ternary phase diagram construction is to demonstrate the proper choice of optimum variety of surfactant and co-surfactant. Depending on the % transmittance, clarity of emulsion, emulsification property PDI and droplet size, F11 formulation was considered optimum and subjected to further characterization [33].

**Fig 8:** Tertiary phase diagram for determining the emulsion region of the SNEDDS.

Twelve (12) formulations containing iodine were prepared. so, all the 12 formulations were analyzed by different characterization techniques like Percentage Transmittance, self-emulsification time, visual observation and thermodynamic stability studies i.e., Centrifugation, Freeze thaw cycle and cloud point measurement. SNEDDS preparation have the capability to encapsulate in nano-emulsion form and also have the capability to solubilize the drug without any drug precipitation or physical instability, such as cracking or creaming. All of the preparations had a size of less than 500 nm, and the poly dispersity index (PDI) values were less than 0.5, like F6 and F11 indicated that they were relatively stable formulations. PDI helps to determine the particles uniformity and its diameter. It is also useful to measure the size distribution of nano-emulsion, which helps to enhance the good particle size distribution. The viscosity of the optimized SNEDDS were determined. The viscosity of F11 was found to be 84.32 ± 1.67 cP. The lesser viscosity of F10 compared to F6 and F11 which may be due to the greater co-surfactant amount. Droplet size distribution have a key part for the evaluation of self nano-emulsifying system. The size of the droplets is thought to be related to drug absorption, as evidenced by earlier research. The smaller as the droplet size of the formulation, more will be the surface area available for drug absorption. The greater antimicrobial impact could be attributed to the lipophilic nature of SNEDDS, which readily interacts with bacteria’s cell membrane to increase iodine interaction when compared to ordinary water iodine. It’s well evaluated that this nano delivery system having lipophilic character having high bacterial cell membrane permeation ability as related with hydrophilic carriers [34]. % Age viability of E. coli in the presence of iodine-containing SNEDDS and unformulated simple iodine at a concentration of 125 g/mL over time. The percentage of iodine released from iodine containing SNEDDS were applied to freshly excised porcine intestinal mucosa. After 3 hours almost 44% of iodine was released from the iodine containing SNEDDS as compared with 95% from unmodified Iodine. By contrast, iodine used as control released almost 90% within an hour as shown in Fig 7.

## Conclusions

Within the scope of this study novel SNEDDS were prepared successfully containing iodine and characterized for size, shape, % transmittance, emulsification properties thermodynamic stability testing, muco- adhesion and enhanced antimicrobial effect. SNEDDS were prepared successfully containing iodine. Selected formulation of SNEDDS showed robust emulsification, size and shape in acceptable range. Muco-penetration and muco-adhesive properties were exhibited by the developed SNEDDS in term of iodine release representing that iodine can reside for longer period in vaginal mucus in comparison to free iodine. SNEDDS containing iodine showed swift and higher antimicrobial activity in comparison to iodine in solution form. Moreover, drug release from SNEDDS was released in 7 hours in slow manner making a viable option for prolong drug release for vaginal cavity. Overall studies showed that iodine in SNEDDS is very effective in comparison to other products available in the market.

## References

[1] KanagalingamJ., et al., Practical use of povidone-iodine antiseptic in the maintenance of oral health and in the prevention and treatment of common oropharyngeal infections. 2015. 69(11): p. 1247–1256.10.1111/ijcp.12707PMC676754126249761

[2] LachapelleJ.-M., et al., Antiseptics in the era of bacterial resistance: a focus on povidone iodine. 2013. 10(5): p. 579.

[3] ZamoraJ.L.J.T.A.j.o.s., Chemical and microbiologic characteristics and toxicity of povidone-iodine solutions. 1986. 151(3): p. 400–406.10.1016/0002-9610(86)90477-03513654

[4] Au-DuongA.-N., LeeC.-K.J.M.S., and E. C, Iodine-loaded metal organic framework as growth-triggered antimicrobial agent. 2017. 76: p. 477–482. doi: 10.1016/j.msec.2017.03.114 28482553

[5] McDonnellG. and RussellA.D.J.C.m.r., Antiseptics and disinfectants: activity, action, and resistance. 2001. 14(1): p. 227.10.1128/cmr.12.1.147PMC889119880479

[6] HeS., et al., Preparation and antimicrobial properties of gemini surfactant-supported triiodide complex system. 2012. 4(4): p. 2116–2123.10.1021/am300094f22404136

[7] DuraniP. and LeaperD.J.I.W.J., Povidone–iodine: use in hand disinfection, skin preparation and antiseptic irrigation. 2008. 5(3): p. 376–387.10.1111/j.1742-481X.2007.00405.xPMC795139518593388

[8] RobinsonJ.R. and BolognaW.J., Vaginal and reproductive system treatments using a bioadhesive polymer, in Advances in Drug Delivery Systems, 6. 1994, Elsevier. p. 87–94.

[9] AhamedM., et al., Facile green synthesis of ZnO-RGO nanocomposites with enhanced anticancer efficacy. Methods, 2021. doi: 10.1016/j.ymeth.2021.04.020 33930572

[10] AhamedM., et al., Facile Synthesis of Zn-Doped Bi2O3 Nanoparticles and Their Selective Cytotoxicity toward Cancer Cells. ACS omega, 2021. 6(27): p. 17353–17361. doi: 10.1021/acsomega.1c01467 34278121PMC8280700

[11] AhamedM., et al., A Novel Green Preparation of Ag/RGO Nanocomposites with Highly Effective Anticancer Performance. Polymers, 2021. 13(19). doi: 10.3390/polym13193350 34641166PMC8512371

[12] KhanK.U., et al., Overview of nanoparticulate strategies for solubility enhancement of poorly soluble drugs. Life Sciences, 2022. 291: p. 120301. doi: 10.1016/j.lfs.2022.120301 34999114

[13] KhanK.U., et al., β-cyclodextrin modification by cross-linking polymerization as highly porous nanomatrices for olanzapine solubility improvement; synthesis, characterization and bio-compatibility evaluation. Journal of Drug Delivery Science and Technology, 2022. 67: p. 102952.

[14] AhamedM., et al., Oxidative stress mediated cytotoxicity and apoptosis response of bismuth oxide (Bi2O3) nanoparticles in human breast cancer (MCF-7) cells. Chemosphere, 2019. 216: p. 823–831. doi: 10.1016/j.chemosphere.2018.10.214 30399561

[15] KhanA.W., et al., Self-nanoemulsifying drug delivery system (SNEDDS) of the poorly water-soluble grapefruit flavonoid Naringenin: design, characterization, in vitro and in vivo evaluation. Drug delivery, 2015. 22(4): p. 552–561. doi: 10.3109/10717544.2013.878003 24512268

[16] AkhterM., et al., Formulation and development of CoQ10-loaded s-SNEDDS for enhancement of oral bioavailability. Journal of Pharmaceutical Innovation, 2014. 9(2): p. 121–131.

[17] ShakeelF., et al., Ultra fine super self-nanoemulsifying drug delivery system (SNEDDS) enhanced solubility and dissolution of indomethacin. Journal of molecular liquids, 2013. 180: p. 89–94.

[18] TalegaonkarS., et al., Design and development of oral oil-in-water nanoemulsion formulation bearing atorvastatin: in vitro assessment. Journal of Dispersion Science and Technology, 2010. 31(5): p. 690–701.

[19] ShafiqS., et al., Development and bioavailability assessment of ramipril nanoemulsion formulation. European journal of pharmaceutics and biopharmaceutics, 2007. 66(2): p. 227–243. doi: 10.1016/j.ejpb.2006.10.014 17127045

[20] BalakumarK., RaghavanC.V., and AbduS., Self nanoemulsifying drug delivery system (SNEDDS) of rosuvastatin calcium: design, formulation, bioavailability and pharmacokinetic evaluation. Colloids and Surfaces B: Biointerfaces, 2013. 112: p. 337–343. doi: 10.1016/j.colsurfb.2013.08.025 24012665

[21] InugalaS., et al., Solid self-nanoemulsifying drug delivery system (S-SNEDDS) of darunavir for improved dissolution and oral bioavailability: in vitro and in vivo evaluation. European Journal of Pharmaceutical Sciences, 2015. 74: p. 1–10. doi: 10.1016/j.ejps.2015.03.024 25845633

[22] DateA.A. and NagarsenkerM., Design and evaluation of self-nanoemulsifying drug delivery systems (SNEDDS) for cefpodoxime proxetil. International journal of pharmaceutics, 2007. 329(1–2): p. 166–172. doi: 10.1016/j.ijpharm.2006.08.038 17010543

[23] ud DinF., et al., Irinotecan-loaded double-reversible thermogel with improved antitumor efficacy without initial burst effect and toxicity for intramuscular administration. Acta biomaterialia, 2017. 54: p. 239–248. doi: 10.1016/j.actbio.2017.03.007 28285074

[24] RizviS.Z.H., et al., Simvastatin-loaded solid lipid nanoparticles for enhanced anti-hyperlipidemic activity in hyperlipidemia animal model. International journal of pharmaceutics, 2019. 560: p. 136–143. doi: 10.1016/j.ijpharm.2019.02.002 30753932

[25] ZidanA.S., et al., Quality by design: Understanding the formulation variables of a cyclosporine A self-nanoemulsified drug delivery systems by Box–Behnken design and desirability function. International journal of pharmaceutics, 2007. 332(1–2): p. 55–63. doi: 10.1016/j.ijpharm.2006.09.060 17169518

[26] SuchaoinW., et al., Development and in vitro evaluation of zeta potential changing self-emulsifying drug delivery systems for enhanced mucus permeation. International Journal of Pharmaceutics, 2016. 510(1): p. 255–262. doi: 10.1016/j.ijpharm.2016.06.045 27329673

[27] AsimM.H., et al., Mucoadhesive S-protected thiolated cyclodextrin-iodine complexes: a promising strategy to prolong mucosal residence time of iodine. Future Microbiology, 2019. 14(5): p. 411–424. doi: 10.2217/fmb-2018-0288 30854897

[28] AhmadJ., et al., Quality by design approach for self nanoemulsifying system of paclitaxel. 2014. 6(8): p. 1778–1791.

[29] WangT., et al., Preparation, quantitive analysis and bacteriostasis of solid state iodine inclusion complex with β-cyclodextrin. 2011. 69(1): p. 255–262.

[30] GursoyR.N., BenitaS.J.B., and pharmacotherapy, Self-emulsifying drug delivery systems (SEDDS) for improved oral delivery of lipophilic drugs. 2004. 58(3): p. 173–182.10.1016/j.biopha.2004.02.00115082340

[31] PoutonC.W. and PorterC.J.J.A.d.d.r., Formulation of lipid-based delivery systems for oral administration: materials, methods and strategies. 2008. 60(6): p. 625–637.10.1016/j.addr.2007.10.01018068260

[32] PorterC.J., et al., Enhancing intestinal drug solubilisation using lipid-based delivery systems. 2008. 60(6): p. 673–691.10.1016/j.addr.2007.10.01418155801

[33] SetthacheewakulS., et al., Development and evaluation of self-microemulsifying liquid and pellet formulations of curcumin, and absorption studies in rats. 2010. 76(3): p. 475–485.10.1016/j.ejpb.2010.07.01120659556

[34] KalepuS., ManthinaM., and PadavalaV.J.A.P.S.B., Oral lipid-based drug delivery systems–an overview. 2013. 3(6): p. 361–372. doi: 10.5005/jp-journals-10024-1445 24858745

